# Mathematical Modeling of Brain Activity under Specific Auditory Stimulation

**DOI:** 10.1155/2021/6676681

**Published:** 2021-04-21

**Authors:** Marius Georgescu, Laura Haidar, Alina-Florina Serb, Daniela Puscasiu, Daniel Georgescu

**Affiliations:** ^1^Functional Sciences Department, Physiology Discipline, Victor Babes University of Medicine and Pharmacy of Timisoara, 2 Eftimie Murgu Sq., Timisoara 300041, Romania; ^2^Biochemistry and Pharmacology Department, Biochemistry Discipline, Victor Babes University of Medicine and Pharmacy of Timisoara, 2 Eftimie Murgu Sq., Timisoara 300041, Romania; ^3^Microscopic Morphology Department, Cellular and Molecular Biology Discipline, Victor Babes University of Medicine and Pharmacy of Timisoara, 2 Eftimie Murgu Sq., Timisoara 300041, Romania; ^4^Functional Disciplines Department, Medical Informatics Discipline, University of Medicine and Pharmacy of Craiova, Craiova 200349, Romania

## Abstract

Understanding the connection between different stimuli and the brain response represents a complex research area. However, the use of mathematical models for this purpose is relatively unexplored. The present study investigates the effects of three different auditory stimuli on cerebral biopotentials by means of mathematical functions. The effects of acoustic stimuli (S1, S2, and S3) on cerebral activity were evaluated by electroencephalographic (EEG) recording on 21 subjects for 20 minutes of stimulation, with a 5-minute period of silence before and after stimulation. For the construction of the mathematical models used for the study of the EEG rhythms, we used the Box-Jenkins methodology. Characteristic mathematical models were obtained for the main frequency bands and were expressed by 2 constant functions, 8 first-degree functions, a second-degree function, a fourth-degree function, 6 recursive functions, and 4 periodic functions. The values obtained for the variance estimator are low, demonstrating that the obtained models are correct. The resulting mathematical models allow us to objectively compare the EEG response to the three stimuli, both between the stimuli itself and between each stimulus and the period before stimulation.

## 1. Introduction

Understanding how the brain functions is one of the utmost scientific challenges of all time. Interdisciplinary research in the fields of neuroscience, physics, biology, neurochemistry, genetics, molecular biology, and psychology has made exciting progress on a wide range of issues. However, as researchers discover evermore functions and locations of brain activity, other scientific concerns arise and no general theory of brain function has been entirely accepted.

Several common techniques exist to measure brain activity: direct imaging techniques—electroencephalography (EEG) and magnetoencephalography (MEG)—which measure electrical or magnetic signal generated due neuronal activity directly and indirect imaging techniques—functional magnetic resonance imaging (fMRI) and positron emission tomography (PET)—which measure neuronal activity using neuronal oxygen consumption. In the case of the EEG and MEG, one joint approach has been to investigate how the time course of brain electrical potentials is influenced by specific stimuli. Combined with controlled sensory stimulation, these methods allow exploration of the sensory and perceptual processes. In this specific area, EEG has been recommended for its non - invasiveness, high temporal resolution, relatively low setup price, possibility of portability and relative ease of use. The influence of different types of external, visual or acoustic, stimuli on cortical EEG has been detailed in various studies [1–8].

Acoustic stimulation through repetitive stimuli, either solely administered or associated with diverse activities can provide new data about complex mental processes [9–11].

Music is a particular type of auditory stimulus because it is a combination of frequency, beat, density, tone, rhythm, repetition, amplitude, and lyrics. Researchers mapped the music-evoked areas of the brain and suggested that music is able to modulate activity in the core areas of emotion, revealing that distinct parts of the brain are activated by music as a function of tonality [12–21].

It has been demonstrated that persistent negative emotional states can increase one's susceptibility to viral infections, yeast infestations, heart attacks, high blood pressure, and other diseases [22]. It is likely that music therapy can influence the autonomous nervous system and reduce stress and stress-related health problems [23], rebalancing the immune system, particularly when the music is known and pleasing to the individual [15, 24, 25]. The effect of music on patients suffering from various neurological disorders or other pathologies has been extensively studied and positive effects have been observed, making music a valuable adjunct to medical practice [26–32].

In addition, classification of emotions based on the EEG while listening to music has currently gained increasing attention due to its potential applications in fields such as music therapy, musical affective brain-computer interface (BCI), neuromarketing, and multimedia tagging and triggering [33].

The profound influence of music training on the functional and structural architecture of auditory-related cerebral areas has been documented by a large number of studies and highlighted the often-observed cognitive advantages of music experts in a variety of cognitive domains, including verbal learning, memory and attention [34–42].

The most noticeable connection between music and increase of performance or altering of neuropsychological activity was shown by studies involving Mozart's music, from which the theory of “The Mozart Effect” [43] was derived. Outcomes of many studies showed that listening to music, especially Mozart compositions (e.g. Mozart sonata K 448) can enhance cognitive performance, motor skills and recovery after brain injury [15, 44–46].

A good part of the EEG studies carried out on Mozart's music showed that listening to Mozart sonata K 448 decreased alpha power which may indicate cortical activation and offer helpful evidence of the Mozart Effect. In addition, significantly decreased EEG theta and beta power were observed [47]. Literature data show that alpha power is regarded as a sensitive indicator of cortical activity and is inversely related to cortical function, decreased values being associated with activations in cortical structures that govern goal-directed cognition and behavior [47, 48]. However, other investigations in this area reported opposite findings, also showing increases in the alpha band in response to music [49, 50]. Despite this, EEG surveys of cerebral activity under acoustic stimulation and, in particular, music, are scarce.

Increased understanding of the relationship between an acoustic stimulus and the brain response will accelerate various researches on the analysis of the brain reaction. Different mathematical and computational methods were used for analysis of the EEG signal under external stimuli [51–56]. Unlike the stereotypical EEG response produced following a short auditory event such as a click or onset of sound, cortical activity associated with continuing stimulation is harder to interpret as responses to each individual event overlap in time, and the lack of repetition prevents simple averaging over trials. Therefore, the development of models from data can be a formidable task, especially in the field of clinical neurophysiology. Thus, several studies focused on characterizing, discriminating or clustering the time series based on the different types of measures applied in preictal EEG segments in order to predict the seizure onset in patients with epilepsy [57–59]. These measures are structured in three main groups: linear, nonlinear, and “other” measures, each group being subdivided in subgroups. The group of linear measures encompasses the subgroups of correlation measures, frequency-based measures and model-based measures. The standard linear models for time series are the autoregressive model (AR) and autoregressive moving average model (ARMA) [60]. Parametric modeling has long been acknowledged as a versatile tool for the analysis of EEG data [61–65].

Modeling of brain activity is a dynamic area of research and several open issues need to be addressed in order to successfully implement these techniques, especially for practical applications such as EEG driven, BCI systems. The potential applications in this direction include BCI-based music recommendation system and BCI-based music therapy, prediction and diagnosis of epilepsy or other neurological impairments. However, literature data on the use of mathematical models in this area is limited.

In this context, our study is aimed at investigating cerebral electrical activity under the influence of different auditory stimuli, both recorded from nature and artificial, different in regard to frequencies, amplitudes, and tonality, by developing, for the first time, mathematical models, in which mathematical functions offer the possibility of study in evolution, with comparisons to the prestimulation period, of the EEG spectral components. Moreover, our data would guide ongoing efforts to develop additional representative models of the brain response to other external stimuli as well as in the case of other brain status.

## 2. Materials and Methods

### 2.1. Subjects

The experiments were carried out in the University of Medicine and Pharmacy of Craiova on 21 males (most of them students), all being right-handed, average age 23 (*σ* = 5.73), without previous musical training, and homogenous regarding professional and extraprofessional activity. Those with a history of neurological disturbances or with a history of drug or ethanol abuse were excluded from the study.

To standardize the group in terms of the degree of fatigue of the subjects, the experiments were performed in the evening, 8 pm, at low levels of noise and natural light.

To select the study group, while ensuring that it is uniform in terms of the perception of sound stimuli, we used a sinusoidal frequency generator coupled to an audio amplifier. The sound provided by the amplifier was perceived by the subjects tested by means of headphones, which were also used in the EEG recording procedure under auditory stimulation. Each subject was subjected to the minimum frequency (45 Hz) at a minimum sound intensity (pressure level). As the subject confirmed the presence of the stimulus, we increased the frequency. When the tested subject signaled the disappearance of the sound stimulus, the intensity was increased up to the limit of 40 dB, which was chosen as the sound intensity level for our study. If the subject did not perceive the sound, he was excluded from the study group. The test ended when we reached the maximum frequency of 16500 Hz. This initial procedure was carried out because the three variants of auditory stimulation we chose encompassed a wide range of frequencies at different intensities.

Starting 12 hours prior to the EEG recording, consumption of none of the following substances—alcohol, caffeine, tea, chocolate, B group vitamins, hormones, hypotensive drugs, sedatives, tranquilizers, sleeping pills—was allowed. Approval for experiments with human subjects for scientific purposes was obtained from The Ethical Commission of the University of Craiova, Romania. Each subject was provided with detailed information about the aims of the ongoing study and gave his written consent to participate in it.

### 2.2. Experimental Stimuli

Auditory stimulation was performed using three different stimuli: S1, an automobile moving on a rough surface, S2, rainfall recorded in a rainforest and S3, two piano sonata K448 by Mozart. The three types of acoustic stimuli were chosen as representative for a monotonous auditory stimulation, subjectively disturbing in case of S1, soothing in case of S2 and pleasant but tensing, in case of S3 [8, 66, 67] (Figure 1).

The three sounds have different characteristics: while in S1 the uniformity of stimulation and the presence of low frequencies are noticeable, with values between 75 Hz and 325 Hz, S2 presents major differences from S1, being much richer in frequencies (the presence of three frequency groups, one below 600 Hz, one around 2000 Hz +/-250 Hz and the last between 3100 and 3800 Hz can be observed), and in variations of amplitudes and tones; while S3 is not a flat, monotonous signal, it is also not quite unpredictable, with repetition intervals which, while not emerging at equal intervals, can still be detected, and a frequency range that is comparable to that of the S2 signal, with some uniform presences distributed.

The EEG was recorded while the subjects were undergoing continuous auditory stimulation, for the duration of 20 minutes, using a pair of headphones (frequency range: 20-20000 Hz) connected to a laptop, powered by its own batteries to avoid parasitic currents. The intensity of the sound was measured with an NM102 Noise Meter and was maintained at a medium level of around 40 dB which was considered safe for the 20 minutes stimulating period in our study activity. We considered the monotony condition to be achieved in stimuli lasting 20 minutes. Longer stimulation periods led to decrease in recording quality, due to the too prolonged discomfort caused by sitting immobile in the chair, electrodes on the scalp, headphones in the ears, or even the reverse – falling asleep.

### 2.3. EEG Recording

The acquisition of cortical biopotentials was made using an industrially produced electroencephalograph, Nihon Kohden EEG-9200. A transformer was used to separate it from the public electricity supply network. The electrodes were placed in the international standard 10–20 system, bipolar acquisition montage, references on the 2 ears, and the extra ECG lead (both hands and the left foot) with the main role of signal quality control.  Figure 2 presents the montage corresponding to the pattern 3 of the collection of cerebral micropotentials.

A great advantage of the Nihon-Kohden EEG-9200 electroencephalograph is that after a bipolar collection, at the time of the acquisition, the data is stored at the sampling rate set initially. This allows adaptation of both the filtration and the collection patterns of the micropotentials according to the requirements of processing. Processing does not affect the original form of the stored data. Spectral analysis can be performed by the program on an artifact-free portion of the EEG, selected by the operator.

During signal inspection, we complied with the requirements of the QP-220AK spectral analysis and mapping program (collection of bipolar brain micropotentials). For a high-fidelity study, the acquisition of signals was made at a high sampling rate (500 Hz), which gives us an EEG that also contains relatively high frequencies (120 Hz), as well as the possibility of performing a Fast Fourier transform (FFT) in the Hanning window on 1024 points for 20 seconds of the signal.

For our study, the frequency band was reduced by more than 60 Hz, and the time constant (the filter passes up) was set to 0.3 s, thus ensuring a sufficiently large bandwidth for the investigated beta, alpha, theta, and delta cerebral rhythms (Table 1).

All recordings were made in identical experimental conditions: subjects with the same degree of physical and psychological tiredness – assessed both subjectively by the examinee and objectively (e.g. number of hours slept previous to experiment) - sitting immobile in a relaxed position, eyes closed, no ambient sound and lighting, no disruptive ambient electrical fields. As an additional measure, a front, grounding electrode was used. The contact impedance during EEG recordings was kept below 30 Kohms and saline solution was used for its reduction, maintaining the contact noise at unanimously acceptable values.

The procedure was carried out as follows—3 valid recordings for each subject, each made under a different stimulus of the three (S1, S2, and S3) (see Figure 3 for the experimental design), with the following well-specified steps:

- Switching on the equipment
- Placement of electrodes and headphones
- Entering the data corresponding to the registration in the EEG program
- Checking the contact impedance and viewing the EEG for control
- Reduction of ambient light
- Start recording
- Subjects close their eyes at the operator's command
- After 5 minutes of silence (L1 period), the operator begins the auditory stimulation
- After 20 minutes of stimulation (S period), the operator stops the auditory stimulation
- After 5 minutes of silence (L2 period), the operator stops the recording
- The operator stores the recording made on the computer
- The subject may open his eyes and be released

To avoid inducing rhythm modulation, subjects were not instructed to follow any particular mental activity, or lack thereof, and were given complete freedom.

Each experiment was carried out in accordance to the general working conditions and the stages inscribed in the protocol, and the recordings performed on the same subject under the influence of auditory stimuli were made on consecutive days (day 1: sound S1, day 2: sound S2, and day 3: sound S3) after 8 pm, in identical working conditions.

After each experiment followed a verification stage, in which the signals were analyzed, for validation, performing repetitions (tests at another time), in case of defective recordings.

### 2.4. EEG Data Processing for Mathematical Modeling

Because our study was limited to the effects of sound stimulation, we only analyzed the data collected from electrodes P3-A1, P4-A2, O1-A1, and O2-A2 (Table 2) by mediation, obtaining a single series of data to characterize the sound projection area.

Following spectral analysis, we subjected data to normalization. Since we are interested in the change of EEG frequencies under external sound stimulation, we compared the values obtained to the normal values of the period without auditory stimulation (the time recorded before the initiation of sound stimulation). We obtained a normalization coefficient for each electrode (average value during the period before stimulation) and, with these values, we applied normalization to each electrode separately (we divided each value recorded by the normalization coefficient).

The mathematical formulas used in the normalization process for the studied derivations are presented below:

(1) $$\begin{array}{c} P3_{ij}^{n}=\frac{P3_{ij}}{1/v-1\sum_{j=1}^{v-1}P3_{ij}}\begin{array}{c} i\in \left\{\text{Delta},\text{Theta},\text{Alpha}1,\text{Alpha}2,\text{Beta}1,\text{Beta}2,\text{Total},\text{Edge},\text{Average},\text{Median},\text{Peak}\right\},\\ j=1,2,\cdots \left(v-1\right),v,\cdots r,\left(r+1\right),\cdots s,\\ v=\text{start stimulation},r=\text{stop stimulation},s=\text{stop acquisition},n=\text{normalized}, \end{array} \end{array}$$

(2) $$\begin{array}{c} P4_{ij}^{n}=\frac{P4_{ij}}{1/v-1\sum_{j=1}^{v-1}P4_{ij}}\begin{array}{c} i\in \left\{\text{Delta},\text{Theta},\text{Alpha}1,\text{Alpha}2,\text{Beta}1,\text{Beta}2,\text{Total},\text{Edge},\text{Average},\text{Median},\text{Peak}\right\},\\ j=1,2,\cdots \left(v-1\right),v,\cdots r,\left(r+1\right),\cdots s,\\ v=\text{start stimulation},r=\text{stop stimulation},s=\text{stop acquisition},n=\text{normalized}, \end{array} \end{array}$$

(3) $$\begin{array}{c} O1_{ij}^{n}=\frac{O1_{ij}}{1/v-1\sum_{j=1}^{v-1}O1_{ij}}\begin{array}{c} i\in \left\{\text{Delta},\text{Theta},\text{Alpha}1,\text{Alpha}2,\text{Beta}1,\text{Beta}2,\text{Total},\text{Edge},\text{Average},\text{Median},\text{Peak}\right\},\\ j=1,2,\cdots \left(v-1\right),v,\cdots r,\left(r+1\right),\cdots s,\\ v=\text{start stimulation},r=\text{stop stimulation},s=\text{stop acquisition},n=\text{normalized}, \end{array} \end{array}$$

(4) $$\begin{array}{c} O2_{ij}^{n}=\frac{O2_{ij}}{1/v-1\sum_{j=1}^{v-1}O2_{ij}}\begin{array}{c} i\in \left\{\text{Delta},\text{Theta},\text{Alpha}1,\text{Alpha}2,\text{Beta}1,\text{Beta}2,\text{Total},\text{Edge},\text{Average},\text{Median},\text{Peak}\right\},\\ j=1,2,\cdots \left(v-1\right),v,\cdots r,\left(r+1\right),\cdots s,\\ v=\text{start stimulation},r=\text{stop stimulation},s=\text{stop acquisition},n=\text{normalized}, \end{array} \end{array}$$

(5) $$\begin{array}{c} M_{ij}^{n}=\frac{1}{4}\cdot \left(P3_{ij}^{n}+P4_{ij}^{n}+O1_{ij}^{n}+O2_{ij}^{n}\right)\begin{array}{c} i\in \left\{\text{D},\text{T},\text{A}1,\text{A}2,\text{B}1,\text{B}2,\text{Total},\text{Edge},\text{Average},\text{Median},\text{Peak}\right\},\\ j=1,2,\cdots s,\\ s=\text{stop acquisition},n=\text{normalized}. \end{array} \end{array}$$

The standardized data series *M*_*ij*_^*n*^ formed the basis for mathematical modeling.

### 2.5. Mathematical Modeling

When building mathematical modeling for the study of the evolution of the total spectrum, as well as for alpha, beta, delta, theta rhythms, we used the Box-Jenkins methodology [68].

In modeling a sample of data as a time series, we searched for patterns in which the process, noted *y*_*t*_, can be described using a white noise process. A stochastic process {*X*_*t*_, *t* ≥ 0} is called white noise if for each *t*, *s* ≥ 0, *X*_*t*_, *X*_*s*_ are uncorrelated, with zero mean and constant dispersion, *σ*^2^.

We will encounter two categories of such time series: autoregressive time series (AR (*p*)) and moving average time series (MA (*q*)).

A *p* order autoregressive time series, (AR (*p*)) is given by the equation: *y*_*t*_ − *θ*_1_*y*_*t*−1_ − *θ*_2_*y*_*t*−2_ − ⋯−*θ*_*p*_*y*_*t*−*p*_ = *a*_*t*_, in which {*a*_*t*_, *t* ≥ 0} is a white noise process.

A time series is a *q* order moving average time series, (MA (*q*)) if given by the equation: *y*_*t*_ = *a*_*t*_ + *φ*_1_*a*_*t*−1_ + *φ*_2_*a*_*t*−2_ + ⋯+*φ*_*q*_*a*_*t*−*q*_.

In addition to these two major categories there are also combined time series, the so-called ARMA (*p*, *q*) models, whose equation is

(6) $$\begin{array}{c} y_{t}-\theta_{1}y_{t-1}-\theta_{2}y_{t-2}-\cdots -\theta_{p}y_{t-p}=a_{t}+\varphi_{1}a_{t-1}+\varphi_{2}a_{t-2}+\cdots +\varphi_{q}a_{t-q}. \end{array}$$

In applications, to find the appropriate serial model for a data sample, a first step is to convert the data series into a series that is similar to an ARMA model. The most commonly applied method is to model the overall trend of the series and the seasonal component, if any. The global trend can be modeled using the regression method. The effective application of the method was made using the program Minitab 16.

The following parameters were used for the modified Box-Pierce (Ljung-Box) Chi-Square statistics: the lag, *p* value, Chi-Square and DF.

The lag represents the time period that separates the data that are ordered in time which is used to calculate the partial autocorrelation coefficient. Minitab displays lags that are in multiples of 12.

The *p* value is a probability that measures the evidence against the null hypothesis. Lower probabilities provide stronger evidence against the null hypothesis.

Chi-square is the test statistic that Minitab uses to determine whether the residuals are independent by calculating the *p* value and comparing the *p* value to the significance level for each chi-square statistic.

DF (the degrees of freedom) represents the amount of information in the presented data, which are used by Minitab program for the chi-square statistics to calculate the *p* value.

The coefficients used for the regression equation/analysis are SE coefficient, *t* value, and *p* value.

SE coefficient (standard error of the coefficient) is used to measure the precision of the estimate of the coefficient. The smaller the standard error, the more precise the estimate. Dividing the coefficient by its standard error a *t* value can be calculated. If the *p* value associated with the *t* statistic is less than the significance level, the coefficient is statistically significant.

The *t* value measures the ratio between the coefficient and its standard error. Minitab uses the *t* value to calculate the *p* value, which is used to test whether the coefficient is significantly different from 0.

Mathematically, the signals obtained from the occipital area were simulated only. This is because the projection in the occipital area is what provides the information for sound perception.

## 3. Results

### 3.1. Delta Rhythm

#### 3.1.1. Mathematical Model in S1 Signal Stimulation

The S1 D time series appears to have a quadratic global trend (Figure 4(a)), which allows for the use of two types of regression models: linear and quadratic, of which the quadratic regression model is the more adequate.

The results of the regression analysis are presented below Table 3:

The regression equation is

(7) $$\begin{array}{c} \text{S}1\text{ D}=0.943701-0.0180543\text{ C}1+0.00114155\text{ C}1*\text{C}1. \end{array}$$

The *p* value of the linear coefficient is marginal (*p* = 0.054), and therefore we decided to retain it, since the quadratic value of the correlation coefficient, *R*^2^ = 48.7%, which reflects the percentage of variation in the S1 D variable, is higher than when the coefficient of the linear term is zero.

We continue the analysis of the residual series, namely the S1 D series, from which we subtracted the regression model. The series is noted below as *z*_*t*_.

Since the coefficient for lag 2 is quite large, the proposed model for the time series *z*_*t*_ is second-order autoregressive, AR (2), of the form

(8) $$\begin{array}{c} z_{t}=\phi_{1}z_{t-1}+\phi_{2}z_{t-2}+a_{t}, \end{array}$$

in which {*a*_*t*_, *t*}  is white noise.

The result for the Box-Jenkins analysis is represented in Tables 4 and 5.

We observed that both coefficients are significant (the *p* values are very low for AR1, AR2) and the *p* value for the Box-Pierce statistics is high, confirming that the {*a*_*t*_, *t*} process can be viewed as being white noise. By combining the result of the regression equation (7) and that of the Box-Jenkins analysis we obtained the model:

(9) $$\begin{array}{c} y_{t}=0.9437-0.0180543t-0.00114155t^{2}+0.4075y_{t-1}-0.6339y_{t-2}+a_{t}. \end{array}$$

#### 3.1.2. Mathematical Model in S2 Signal Stimulation

The S2 D series is represented in Figure 4(b). The global trend is linear and ascending, and also presents a somewhat periodic behavior, for which it is difficult to define the period, which is why we used a linear regression. The regression equation is

(10) $$\begin{array}{c} {\hat{y}}_{t}=0.8072+0.0607t. \end{array}$$

If we subtract from the S2 D series the model given by equation (10), we obtain the series RESI7, represented in the graph in Figure 4(c).

Next, we model the seasonal component of the series, using a trigonometric function:

(11) $$\begin{array}{c} {\hat{y}}_{t}=0.3\sin\left(\left(t-11\right)\frac{\pi }{4}\right). \end{array}$$

The RESI7 series, together with the model proposed in equation (11) are represented in Figure 4(d). The pattern given by equation (11) is represented in red in the graphical expression.

We noted the residuals of the RESI7 series after the elimination of the sinusoidal model as RESI9.

Thus, the model found by this method is

(12) $$\begin{array}{c} y_{t}=0.8072+0.0607t+0.3\sin\left(\left(t-11\right)\frac{\pi }{4}\right)+a_{t}. \end{array}$$

We estimate the variance of white noise as being ${\overset{\wedge }{\sigma }}^{2}\left(y_{t}\right)={\overset{\wedge }{\sigma }}^{2}\left(a_{t}\right)=0.1642$.

#### 3.1.3. Mathematical Model in S3 Signal Stimulation

Although the graph of the S3 D series appears to show the global quadratic trend (see Figure 4(e)), we opted to use a linear model, because the quadratic model had a non-significant second-order coefficient.

For the modeling of residuals, we chose a 1st-order moving average, MA (1).

The obtained model is significant, the autocorrelation and partial autocorrelation functions show that the model is suitable and an advantage of such a model is that it was obtained with a minimum number of parameters (coefficients).

In conclusion, the model obtained is

(13) $$\begin{array}{c} y_{t}=1.18+0.021t+a_{t}-0.9033a_{t-1}. \end{array}$$

### 3.2. Theta Rhythm

#### 3.2.1. Mathematical Model in S1 Signal Stimulation

The time series S1 theta (T) has an ascending global trend (see Figure 5(a)), with a slight increase in variance and without a seasonal component, which is why the most suitable option for modeling is to use a second-degree polynomial function, with the following equation:

(14) $$\begin{array}{c} y_{t}=0.95+0.00051t^{2}+a_{t}, \end{array}$$

in which we can estimate the variance of white noise ${\overset{\wedge }{\sigma }}^{2}\left(y_{t}\right)={\overset{\wedge }{\sigma }}^{2}\left(a_{t}\right)=0.0073.$

#### 3.2.2. Mathematical Model in S2 Signal Stimulation

The S2 T time series (Figure 5(b)) has an ascending, linear global trend, without seasonal component. The proposed model for S2 T is

(15) $$\begin{array}{c} y_{t}=0.9622+0.0186t+a_{t}. \end{array}$$

The estimated value for the white noise process variant is

(16) $$\begin{array}{c} {\overset{\wedge }{\sigma }}^{2}\left(y_{t}\right)={\overset{\wedge }{\sigma }}^{2}\left(a_{t}\right)=0.0218. \end{array}$$

#### 3.2.3. Mathematical Model in S3 Signal Stimulation

The S3 T time series has an ascending, linear global trend, with a tendency for the variance to increase. The series also seems to have a seasonal composition, of period 6 (Figure 5(c)).

We transformed the series to transform it into a constant variance series.

Usually, the transformation that is used in such cases is a power function. In this case we used the following transformation:

(17) $$\begin{array}{c} x_{t}=y_{t}^{1/4}, \end{array}$$

where *y*_*t*_ represents the original data series, S3 T.

Next, we modeled the global trend of the series with a linear model:

(18) $$\begin{array}{c} {\hat{x}}_{t}=0.971+0.00655t. \end{array}$$

The graph of the residuals obtained following the elimination of the global trend (named RESI6) is presented in Figure 5(d).

The pattern found for the residue series is a first-order seasonal moving average (SMA (1)): *z*_*t*_ = *a*_*t*_ − *θa*_*t*−6_ .

The results of the analysis are presented in Tables 6 and 7.

We observed that the *p* value for the model coefficient is small; thus, the coefficient is significant.

On the other hand, the *p* value for the Box-Pierce statistics is high, confirming that the residual process can be seen as white noise.

The model found for S3 T is

(19) $$\begin{array}{c} y_{t}={\left(0.971+0.00655t+a_{t}+0.733a_{t-6}\right)}^{4}, \end{array}$$

### 3.3. Alpha Rhythm

#### 3.3.1. Mathematical Model for Alpha 1 Rhythm in S1 Signal Stimulation

The S1 alpha 1 (A1) series is graphically represented in Figure 6(a).

We observed that the series has an approximately constant global trend and also seems to have a seasonal component of period 6. Calculating the slope of the regression line, we found it to be non-significant (*p* = 0.35). This fact led us to the proposal of a regression line, which would be constant,$\;{\hat{y}}_{t}=0.727$ (the value of the constant is the average of the S1 A1 series).

The indexes of the seasonal component, identified using the Minitab software, are the following:

*c*_1_ = 0.142, *c*_2_ = 0.023, *c*_3_ = −0.041, *c*_4_ = −0.068, *c*_5_ = −0.135, *c*_6_ = 0.025.

The residuals of the model thus constructed have the appearance of a white noise process (which is confirmed by the graphs of the autocorrelation and partial autocorrelation functions), so the proposed model for the S1 A1 series is

(20) $$\begin{array}{c} y_{t}=0.727+c_{t\left(\mathrm{mod}6\right)}+a_{t}, \end{array}$$

where *t*(mod6) is the value of the remainder of dividing *t* by 6. The estimated value for the white noise process variant is

(21) $$\begin{array}{c} {\overset{\wedge }{\sigma }}^{2}\left(y_{t}\right)={\overset{\wedge }{\sigma }}^{2}\left(a_{t}\right)=0.0158. \end{array}$$

#### 3.3.2. Mathematical Model for Alpha 1 Rhythm in S2 Signal Stimulation

The S2 A1 time series has an ascending, linear global trend, without a seasonal component (Figure 6(b)). The model constructed with linear regression is ${\hat{y}}_{t}=0.688+0.007t$; however, the *p* for the slope of the line is marginally non-significant (*p* = 0.056).

The second model we tested is a constant line in which the value of the constant is the average of the series S2 A1: ${\hat{y}}_{t}=0.764$. The residuals obtained with this global trend model present functions of autocorrelation and partial autocorrelation corresponding to a white noise process, and therefore we can model the S2 A1 series: *y*_*t*_ = 0.764 + *a*_*t*_ in which the variance of the white noise process is estimated to be ${\overset{\wedge }{\sigma }}^{2}\left(y_{t}\right)={\overset{\wedge }{\sigma }}^{2}\left(a_{t}\right)=0.099$

#### 3.3.3. Mathematical Model for Alpha 1 Rhythm in S3 Signal Stimulation

The S3 A1 series is presented in Figure 6(c). We observed an ascending trend, possibly quadratic, with a slight increase in variance. A seasonal component is possible; however, the period is difficult to define.

A first attempt to model the global trend, through a second-degree polynomial, demonstrates that such a model is non-significant, since the coefficients have very high *p* values. A second attempt was to consider the series of first-order differences: *x*_*t*_ = *y*_*t*_ − *y*_*t*−1_, *t* ≥ 1, the graph of which is presented in Figure 6(d).

We observed that the series has a constant global trend; the variance appears to be constant and does not appear to have a seasonal component. An analysis of the autocorrelation and partial autocorrelation functions suggests a first-order moving average model, MA (1): *x*_*t*_ = *a*_*t*_ − *θa*_*t*−1_, *t* ≥ 1. The result of the Box-Jenkins analysis is presented below. The model coefficient is significant and the model is adequate, as shown by the *p* value for the Box-Pierce statistics Tables 8 and 9.

Also to be considered is that the graphs of the autocorrelation and partial autocorrelation functions of the model residuals confirms that the residuals are a white noise process. We conclude that an appropriate model is

(22) $$\begin{array}{c} y_{t}-y_{t-1}=a_{t}-0.71a_{t-1}. \end{array}$$

Estimating the variance of the white noise process is ${\overset{\wedge }{\sigma }}^{2}\left(a_{t}\right)={\overset{\wedge }{\sigma }}^{2}\left(y_{t}-y_{t-1}\right)/\left(1+0.71^{2}\right)=0.0542/1+0.71^{2}=0.036$.

#### 3.3.4. Mathematical Model for Alpha 2 Rhythm in S1 Signal Stimulation

The S1 A2 series has an almost constant global trend, without seasonal component; however, we did observe a sudden drop at time *t* = 13 (Figure 7(a)).

We used a linear regression model for the global trend of the series:

(23) $$\begin{array}{c} y_{t}=1.106-0.021t+a_{t}. \end{array}$$

We estimate the variance of the white noise process as

(24) $$\begin{array}{c} {\overset{\wedge }{\sigma }}^{2}\left(y_{t}\right)={\overset{\wedge }{\sigma }}^{2}\left(a_{t}\right)=0.1943. \end{array}$$

#### 3.3.5. Mathematical Model for Alpha 2 Rhythm in S2 Signal Stimulation

The S2 A2 series has a quadratic global trend, with an ascending variance, and appears to have a seasonal appearance (Figure 7(b)); however, the data is insufficient to confirm whether the pattern is repeated periodically or not.

We transformed the series, taking into account the first-order differences, and thus define the new series as *x*_*t*_ = *y*_*t*_ − *y*_*t*−1_, *t* ≥ 1 (Figure 7(c)).

We observed that the series seems to present constant variance. A model of first-order seasonal moving average (with period 4, SMA 4) produces the result shown in Tables 10 and 11.

The model coefficient is significant, and the Box-Pierce statistics show that the model has residuals that may belong to a white noise process (*p* = 0.25). We therefore conclude that a plausible model for the S2 A2 series is

(25) $$\begin{array}{c} y_{t}-y_{t-1}=a_{t}-0.822a_{t-4}. \end{array}$$

We can estimate the variance of the white noise process:

(26) $$\begin{array}{c} {\overset{\wedge }{\sigma }}^{2}\left(a_{t}\right)=\frac{{\overset{\wedge }{\sigma }}^{2}\left(y_{t}-y_{t-1}\right)}{1+0.822^{2}}=\frac{0.032}{1+0.822^{2}}=0.019. \end{array}$$

#### 3.3.6. Mathematical Model for Alpha 2 Rhythm in S3 Signal Stimulation

The S3 A2 series appears to have a global tendency similar to a sinusoid, with an approximately constant variance, without the seasonal component (Figure 7(d)).

After transforming the series, and considering the first-order differences, we obtained a series which can be interpreted as a white noise process (Figure 7(e)).

Thus, a plausible model is *y*_*t*_ − *y*_*t*−1_ = *a*_*t*_, with the white noise variant estimated as being ${\overset{\wedge }{\sigma }}^{2}\left(a_{t}\right)={\overset{\wedge }{\sigma }}^{2}\left(y_{t}-y_{t-1}\right)=0.074$.

### 3.4. Beta Rhythm

#### 3.4.1. Mathematical Model for Beta 1 Rhythm in S1 Signal Stimulation

The series has an overall decreasing trend, without a seasonal component (Figure 8(a)). By linear regression, we modeled the global trend with a line:

(27) $$\begin{array}{c} {\hat{y}}_{t}=0.967-0.0077t. \end{array}$$

The result of the regression analysis shows that both coefficients are significant Table 12.

The regression equation is

(28) $$\begin{array}{c} \text{S}1\text{ B}1=0.967-0.00768\text{ C}1. \end{array}$$

After eliminating the global trend, the residuals obtained have autocorrelation and partial autocorrelation functions graphs which can be interpreted as belonging to a white noise process. Thus, we can model the S1 B1 series as *y*_*t*_ = 0.967 − 0.0077*t* + *a*_*t*_ with the white noise variance estimated to be ${\overset{\wedge }{\sigma }}^{2}\left(a_{t}\right)={\overset{\wedge }{\sigma }}^{2}\left(y_{t}\right)=0.0054$.

#### 3.4.2. Mathematical Model for Beta 1 Rhythm in S2 Signal Stimulation

The S2 B1 series has an ascending global trend, with a seasonal component of period 6, which is presented in Figure 8(b).

The equation for the global trend was obtained by linear regression:

(29) $$\begin{array}{c} {\hat{y}}_{t}=0.8234+0.0102t. \end{array}$$

The seasonal component of period 6 has the following values:

(30) $$\begin{array}{c} c_{1}=-0.0726,c_{2}=-0.0181,c_{3}=0.0635,c_{4}=-0.0678,c_{5}=-0.0182,c_{6}=-0.0181. \end{array}$$

The original series, together with the model given by the global trend and the seasonal component, are represented in Figure 8(c).

The residuals series has the characteristics of a white noise process, and thus, we can conclude that the model of the series is

(31) $$\begin{array}{c} y_{t}=0.8234+0.0102t+c_{t\left(\mathrm{mod}6\right)}+a_{t},{\overset{\wedge }{\;\sigma }}^{2}\left(a_{t}\right)={\overset{\wedge }{\sigma }}^{2}\left(y_{t}\right)=0.0074. \end{array}$$

#### 3.4.3. Mathematical Model for Beta 1 Rhythm in S3 Signal Stimulation

The series has an ascending global trend, with a slight increase in variance which is difficult to verify, given the size of the data sample (Figure 8(d)).

The global trend can be modeled using a linear regression:

(32) $$\begin{array}{c} {\hat{y}}_{t}=0.8047+0.016t. \end{array}$$

After eliminating the global trend, the residuals series can be seen as a white noise process, so a suitable model for the series is

(33) $$\begin{array}{c} y_{t}=0.805+0.016t+a_{t}{\overset{\wedge }{\sigma }}^{2}\left(a_{t}\right)={\overset{\wedge }{\sigma }}^{2}\left(y_{t}\right)=0.0172. \end{array}$$

#### 3.4.4. Mathematical Model for Beta 2 Rhythm in S1 Signal Stimulation

In Figure 9(a) we present the evolution in time of the series of values corresponding to the beta 2 rhythm, under auditory stimulation with the S1 signal. This series (S1 B2) has a decreasing global trend, without a seasonal component. As a global trend model, we propose the linear regression line: ${\hat{y}}_{t}=1.04-0.0067t$.

The series of residuals obtained, after we subtracted the linear model, RESI13, appears to be a white noise process, although an analysis of the autocorrelation and partial autocorrelation functions shows an increase of the values of the autocorrelation coefficients with the increase of the gap (although the values remain in the 95% confidence band).

Given that we used a fairly short range of values, it is difficult to establish how the autocorrelation function behaves at larger gaps. Thus, a first model that we propose is

(34) $$\begin{array}{c} y_{t}=1.04-0.0067t+a_{t},{\overset{\wedge }{\sigma }}^{2}\left(a_{t}\right)={\overset{\wedge }{\sigma }}^{2}\left(y_{t}\right)=0.079, \end{array}$$

A second model we propose is the following: first we consider the series of first-order differences. Then, since the lag 1 autocorrelations coefficients were high and then decreased sharply, a first-order moving average model, MA (1) is advised.

The model is

(35) $$\begin{array}{c} y_{t}-y_{t-1}=a_{t}-0.81a_{t-1},{\overset{\wedge }{\sigma }}^{2}\left(a_{t}\right)=\frac{{\overset{\wedge }{\sigma }}^{2}\left(y_{t}-y_{t-1}\right)}{1+0.81^{2}}=\frac{0.0123}{1+0.81^{2}}=0.0074. \end{array}$$

#### 3.4.5. Mathematical Model for Beta 2 Rhythm in S2 Signal Stimulation

The S2 BS series is represented in Figure 9(b).

We distinguish an ascending global trend, with a seasonal character of period 6. The equation for the global trend was obtained by a linear regression:

(36) $$\begin{array}{c} {\hat{y}}_{t}=0.8833+0.0038t. \end{array}$$

The seasonal component of period 6 has the following values:  *c*_1_ = −0.0543, *c*_2_ = 0.0054, *c*_3_ = 0.0152, *c*_4_ = 0.0686, *c*_5_ = 0.0004, and *c*_6_ = −0.0393.

The original series, together with the model, are represented in Figure 9(c). The series of residuals has the characteristics of a white noise process; we can decide that the series model is

(37) $$\begin{array}{c} y_{t}=0.8833+0.0038t+c_{t\left(\mathrm{mod}6\right)}+a_{t},{\overset{\wedge }{\sigma }}^{2}\left(a_{t}\right)={\overset{\wedge }{\sigma }}^{2}\left(y_{t}\right)=0.0038. \end{array}$$

#### 3.4.6. Mathematical Model for Beta 2 Rhythm in S3 Signal Stimulation

The S3 B2 series is very similar to the S3 B1 series: the same sudden increase is observed at the 16th value in the series. Beyond this, the series seems to have a decreasing global trend, without a seasonal aspect (Figure 9(d)). The equation given by linear regression is

(38) $$\begin{array}{c} {\hat{y}}_{t}=0.888+0.007t. \end{array}$$

The Box-Jenkins analysis shows that the MA (2) model is adequate: the coefficients have very low *p* values and that the *p* value for the Box-Pierce statistic is high Tables 13 and 14.

We can thus decide that the S3 B2 series model is

(39) $$\begin{array}{c} y_{t}=0.888+0.007t+a_{t}+1.0622a_{t-1}+0.8a_{t-2},\\ {\overset{\wedge }{\sigma }}^{2}\left(a_{t}\right)=\frac{{\overset{\wedge }{\sigma }}^{2}\left(y_{t}\right)}{1+1.0622^{2}+0.8^{2}}=\frac{0.0184}{2.7683}=0.0066. \end{array}$$

## 4. Discussion

In this paper, we estimated the variance from the residuals of the mean fit to each signal series. Therefore, the smaller the estimate for the variance, the better the regression fit to the series. Following the values of the obtained models, we obtained a sufficiently small variance size – with the exception of three cases in which a value could not be obtained.

The resulting mathematical functions offer the possibility to study, during the 20 minutes of stimulation, the evolution in time, compared to the period prior to stimulation, of the spectral composition of the EEG.

In Table 15 the mathematical models of the alpha, beta, delta and theta rhythms corresponding to the S1 sound are presented.

We observe that the alpha rhythm (A1 and A2) has the largest variance, and generally the lowest amplitude while the theta rhythm has the highest amplitude, at least towards the end of the period when the S1 stimulation was applied. Indeed, the mean values of the alpha waves (Table 16) are among the lowest (0.727 for alpha1 and 0.889 for alpha2), while the mean value of the theta wave is 1.023. Also, the amplitude of the theta waves tends to increase towards the end of the period when the S1 stimulus was applied, reaching the value of about 1.2, compared to the minimum amplitude of about 0.55, reached by the alpha1 wave.

Regarding the S2 sound, (Table 17) the alpha waves again show the lowest amplitude, while the delta rhythm has the highest amplitude and increasing in the second half of the period when the sound was applied, reaching up to a value of about 2.15. Analyzing the standard deviations from Table 18, the delta rhythm has the highest value (0.405), while the smallest deviation is the beta2 wave (0.062). We also notice that the beta1 and beta2 frequency bands are almost identical, a fact confirmed by the similarity of the two models found by the Box-Jenkins analysis.

The graphs show the greatest separation between the S2 sound when compared to the S1 sound.

Mathematical models for brain rhythms corresponding to S3 stimulation are given in Table 19. As with the S2 stimulus, delta and theta rhythms appear to dominate in the second half of the time interval. It is interesting to note in Table 20 that the standard deviations are mostly close to 0.2, except for the beta1 and beta2 frequency bands which have values close to 0.13.

If we compare the results obtained after the stimulation with the three types of complex sounds, grouping by frequency band, we notice that for both the alpha1 and alpha2 frequency bands the lowest average values (0.727 and 0.889, respectively) are recorded for the S1 stimulus and the highest mean values are for the S3 stimulus (0.901 and 1.027, respectively). In terms of standard deviation, it is higher for S3 sound for both alpha1 and alpha2 waves.

For the beta rhythm, the mean values are much closer than in the case of alpha waves ranging between 0.8859 (S1 B1) and 0.9726 (S3 B1). Standard deviations are also lower, ranging from 0.0733 (S1 B1) to 0.1357 (S3 B2). Thus, S3 for beta1 has the highest average on the considered interval for beta 2, while the sound S1 has the highest average, slightly exceeding S3.

The delta rhythm shows a much more interesting behavior: the average values increase from 0.9179 for the S1 sound to 1.4445 for the S2 sound and 1.3981 for the S3 sound. Standard deviations also increase significantly, from 0.07 for S1 to 0.405 for S2 and 0.2027 for S3. A clear domination of the waves corresponding to the signals S2 and S3 is observed.

The same increase is observed for the theta rhythm: the average values increase from 1.0232 for S1 to 1.183 for the S3 stimulus, but the increase is much smaller than that recorded for delta or alpha rhythms. The theta rhythm corresponding to the sounds S2 and S3 dominates the one corresponding to S1. The standard deviation is as in the case of the other studied rhythms higher for S2 and S3 (0.1477 and 0.2019, respectively) compared to 0.0852 for S1.

## 5. Conclusions

In the present study, a model was obtained for the th5ree types of stimulation signals S1, S2, and S3 which generated mathematical functions for the main waves of the electroencephalogram: alpha, beta, delta, and theta. Mathematical models give us the possibility to compare simply but objectively the response of the encephalogram to the stimuli S1, S2, and S3.

Synthetically, mathematical models were obtained expressed by 2 constant functions, 8 first-degree functions (linear), a second-degree function, a fourth-degree function, 6 recursive functions, and 4 periodic functions.

Each sound stimulation produced a characteristic pattern of changes in cortical micropotentials: S3 predominantly influences the low-frequency bands (for theta *p* = 0.003), S1 influences those of higher frequencies (for beta *p* = 0.027), and S2 exerts a moderate influence on both bands, with a slight predominance over the low-frequency ones.

In most models for the residuals, the estimate for the variance is rather small, indicating that the signal series can be modeled quite accurately.

The resulting mathematical functions offer the possibility of studying, for the 20 stimulation minutes, of the evolution in time, compared to the period before stimulation, of the EEG spectral component.

The development of a mathematical model which allows the study of evolution of the spectral EEG component represents an aspect of originality of this study and marks the practical importance, in the case of monotonous auditory stimulations, of the interval of time in which the synchronization of cerebral activity, depending on the type of stimulation, may occur.

## Figures and Tables

**Figure 1:** Graph of the sound amplitude over time for the three acoustic stimuli: (a) S1, (b) S2, (c) and S3.

**Figure 2:** Collection pattern of the cerebral micropotentials.

**Figure 3:** Overview of the experimental workflow.

**Figure 4:** Graphs of the delta (D) series: (a) time function graph of the S1 D series values; (b) time function graph of the S2 D series values; (c) graph of the RESI7 series corresponding to S2 D; (d) graphs of the RESI7 series and the sinusoidal model corresponding to S2 D; (e) time function graph of the S3 D series values.

**Figure 5:** Graphs of the theta (T) series: (a) time function graph of the S1 T series values; (b) time function graph of the tendency (trend) and of the model of S2 T series; (c) time function graph of the S3 T series values; (d) graph of the RESI6 series corresponding to S3 T. MAPE: the mean absolute percent error; MAD: the mean absolute deviation; MSD: the mean square deviation.

**Figure 6:** Graphs of the alpha 1 (A1) series: (a) time function graph of the S1 A1 series values; (b) time function graph of the S2 A1 series values; (c) time function graph of the S3 A1 series values; (d) the first-order difference graph for the S3 A1 series.

**Figure 7:** Graphs of the alpha 2 (A2) series: (a) the time function graph of the S1 A2 series values; (b) the time function graph of the S2 A2 series values; (c) the first-order difference graph for the S2 A2 series; (d) the time function graph of the S3 A2 series values; (e) the first-order difference graph for the S3 A2 series.

**Figure 8:** Graphs of the beta 1 (B1) series: (a) time function graph of the S1 B1 series values; (b) time function graph of the S2 B1 series values; (c) time function graph of the tendency (trend) and of the model of S2 B1 series; (d) time function graph of the S3 B1 series values. MAPE: the mean absolute percent error; MAD: the mean absolute deviation; MSD: the mean square deviation.

**Figure 9:** Graphs of the beta 2 (B2) series: (a) the time function graph of the S1 B2 series values; (b) the time function graph of the S2 B2 series values; (c) the time function graph of the tendency (trend) and of the model of S2 B2 series; (d) the time function graph of the S3 B2 series values. MAPE: the mean absolute percent error; MAD: the mean absolute deviation; MSD: the mean square deviation.

**Table 1:** Brain rhythms separated by the QP-220AK program.

EEG rhythm	Frequency band (Hz)	The filter passes up (Hz)	The filter passes down (Hz)
Delta	2-4	2	4
Theta	4-8	4	8
Alpha 1	8-10	8	10
Alpha 2	10-13	10	13
Beta 1	13-20	13	20
Beta 2	20-30	20	30

**Table 2:** Data provided by the encephalograph following spectral analysis (for an EEG segment of 20 sec).

		Median value for EEG rhythms							Indices for the whole spectrum			
		Delta	Theta	Alpha 1	Alpha 2	Beta 1	Beta 2	Total	Edge	Av	Median	Peak
P3	A1	2.766	2.8	4.785	3.615	2.088	1.515	17.568	19.141	10.16	9.57	10.16
P4	A2	3.727	3.78	6.639	3.854	1.521	0.783	20.304	13.672	8.789	9.18	10.16
O1	A1	2.257	2.971	13.644	16.39	2.591	1.895	39.745	14.453	10.35	9.961	10.16
O2	A2	2.416	4.028	13.17	13.79	1.93	1.398	36.729	11.914	9.961	9.961	10.16

Edge (edge frequency): the frequency that establishes, at a value initially set by the operator (90% in our case), the ratio—the left area/the whole area of the spectrum; Av (average frequency): the frequency corresponding to the center of gravity of the spectrum area; median (median frequency): the frequency that divides the area into two equal parts; peak (peak frequency): the maximum energy frequency.

**Table 3:** Coefficients.

Term	Coef	SE coef	*T*	*P*
Constant	0.943701	0.0397789	23.7236	0.001
C1	-0.018054	0.0087241	-2.0695	0.054
C1∗C1	0.001142	0.0004035	2.8289	0.012

**Table 4:** Final estimation of parameters.

Type	Coef	SE coef	*T*	*P*
AR 1	0.4075	0.1823	2.24	0.038
AR 2	-0.6339	0.1823	-3.48	0.003

**Table 5:** Modified Box-Pierce (Ljung-Box) chi-square statistics.

Lag	12	24	36	48
Chi-square	8.8	∗	∗	∗
DF	10	∗	∗	∗
*P*	0.549	∗	∗	∗

**Table 6:** Final estimation of parameters.

Type	SE coef	Coef	*T*	*P*
SMA 6	-0.7330	0.2948	-2.49	0.022

**Table 7:** Modified Box-Pierce (Ljung-Box) chi-square statistics.

Lag	12	24	36	48
Chi-square	11.8	∗	∗	∗
DF	11	∗	∗	∗
*P*	0.376	∗	∗	∗

**Table 8:** Final estimation of parameters.

Type	Coef	SE coef	*T*	*P*
MA 1	0.7101	0.1887	3.76	0.001

**Table 9:** Modified Box-Pierce (Ljung-Box) chi-square statistics.

Lag	12	24	36	48
Chi-square	10.5	∗	∗	∗
DF	11	∗	∗	∗
*P*	0.483	∗	∗	∗

**Table 10:** Final estimation of parameters.

Type	Coef	SE coef	*T*	*P*
SMA 4	0.8219	0.2150	3.82	0.001

**Table 11:** Modified Box-Pierce (Ljung-Box) chi-square statistics.

Lag	12	24	36	48
Chi-square	13.7	∗	∗	∗
DF	11	∗	∗	∗
*P*	0.250	∗	∗	∗

**Table 12:** 

	Coef	SE coef	*T*	*P*
Constant	0.96655	0.02746	35.19	0.001
C1	-0.007679	0.002293	-3.35	0.004

**Table 13:** Final estimation of parameters.

Tip	Coef	SE coef	*T*	*P*
MA 1	-1.0622	0.2281	-4.66	0.001
MA 2	-0.8011	0.2220	-3.61	0.002

**Table 14:** Modified Box-Pierce (Ljung-Box) chi-square statistics.

Lag	12	24	36	48
Chi-square	5.3	∗	∗	∗
DF	10	∗	∗	∗
*P*	0.869	∗	∗	∗

**Table 15:** Comparative presentation of mathematical models in the case of S1 stimulation.

EEG spectrum	Mathematical model	Variance estimator ${\overset{\wedge }{\sigma }}^{2}\left(a_{t}\right)$
Delta	*y*_*t*_ = 0.9437 − 0.0180543*t* − 0.00114155*t*^2^ + 0.4075*y*_*t*−1_ − 0.6339*y*_*t*−2_ + *a*_*t*_	
Theta	*y*_*t*_ = 0.95 + 0.00051*t*^2^ + *a*_*t*_	0.0073
Alpha 1	*y*_*t*_ = 0.727 + *c*_*t*(mod6)_ + *a*_*t*_ *c*_1_ = 0.142, *c*_2_ = 0.023, *c*_3_ = −0.041, *c*_4_ = −0.068, *c*_5_ = −0.135, *c*_6_ = 0.025	0.0158
Alpha 2	*y*_*t*_ = 1.106 − 0.021*t* + *a*_*t*_	0.1943
Beta 1	*y*_*t*_ = 0.967 − 0.0077*t* + *a*_*t*_	0.054
Beta 2	*y*_*t*_ = 1.04 − 0.0067*t* + *a*_*t*_	0.079

**Table 16:** Statistical analysis of the values generated in the case of stimulation with the S1 signal.

	*N*	Average	Standard deviation	Minimum	Q1	Median	Q3	Maximum
S1 A1	20	0.7270	0.1256	0.5418	0.6369	0.6928	0.8359	1.0130
S1 A2	20	0.8894	0.1943	0.5973	0.7056	0.9512	1.0671	1.1849
S1 B1	20	0.8859	0.0733	0.7710	0.8057	0.8989	0.9501	1.0026
S1 B2	20	0.9655	0.0890	0.8055	0.9053	0.9582	1.0291	1.1430
S1 D	20	0.9179	0.0706	0.7861	0.8788	0.9161	0.9624	1.0648
S1 T	20	1.0232	0.0852	0.9281	0.9655	0.9904	1.0703	1.1992

**Table 17:** Comparative presentation of mathematical models in the case of S2 stimulation.

EEG spectrum	Mathematical model	Variance estimator ${\overset{\wedge }{\sigma }}^{2}\left(a_{t}\right)$
Delta	$y_{t}=0.8072+0.0607t+0.3\sin\left(\left(t-11\right)\frac{\pi }{4}\right)+a_{t}$	0.1642
Theta	*y*_*t*_ = 0.9622 + 0.0186*t* + *a*_*t*_	0.0218
Alpha 1	*y*_*t*_ = 0.764 + *a*_*t*_	0.099
Alpha 2	*y*_*t*_ − *y*_*t*−1_ = *a*_*t*_ − 0.822*a*_*t*−4_	0.019
Beta 1	*y*_*t*_ = 0.8234 + 0.0102*t* + *c*_*t*(mod6)_ + *a*_*t*_ *c*_1_ = −0.0726, *c*_2_ = −0.0181, *c*_3_ = 0.0635, *c*_4_ = −0.0678, *c*_5_ = −0.0182, *c*_6_ = −0.0181	0.074
Beta 2	*y*_*t*_ = 0.8833 + 0.0038*t* + *c*_*t*(mod6)_ + *a*_*t*_ *c*_1_ = −0.0543, *c*_2_ = 0.0054, *c*_3_ = 0.0152, *c*_4_ = 0.0686, *c*_5_ = 0.0004, *c*_6_ = −0.0393.	0.038

**Table 18:** Statistical analysis of the values generated in the case of stimulation with the S2 signal.

	*N*	Average	Standard deviation	Minimum	Q1	Median	Q3	Maximum
S2 A1	20	0.7640	0.0988	0.6129	0.7118	0.7404	0.8421	0.9440
S2 A2	20	0.9150	0.1913	0.5319	0.7707	0.9289	1.0382	1.2770
S2 B1	20	0.9255	0.0823	0.8165	0.8616	0.9166	0.9727	1.0946
S2 B2	20	0.9236	0.0620	0.8311	0.8808	0.9202	0.9575	1.1015
S2 D	20	1.4445	0.4053	0.8183	1.0530	1.4260	1.7606	2.1503
S2 T	20	1.1575	0.1477	0.8869	1.0406	1.1780	1.2582	1.4131

**Table 19:** Comparative presentation of mathematical models in the case of S3 stimulation.

EEG spectrum	Mathematical model	Variance estimator ${\overset{\wedge }{\sigma }}^{2}\left(a_{t}\right)$
Delta	*y*_*t*_ = 1.18 + 0.021*t* + *a*_*t*_ − 0.9033*a*_*t*−1_	0.0226
Theta	*y*_*t*_ = (0.971 + 0.00655*t* + *a*_*t*_ + 0.733*a*_*t*−6_)^4^	—
Alpha 1	*y*_*t*_ − *y*_*t*−1_ = *a*_*t*_ − 0.71*a*_*t*−1_	0.036
Alpha 2	*y*_*t*_ − *y*_*t*−1_ = *a*_*t*_	0.074
Beta 1	*y*_*t*_ = 0.805 + 0.016*t* + *a*_*t*_	0.0172
Beta 2	*y*_*t*_ = 0.888 + 0.007*t* + *a*_*t*_ + 1.0622*a*_*t*−1_ + 0.8*a*_*t*−2_	0.0066

**Table 20:** Statistical analysis of the values generated in the case of stimulation with the S3 signal.

	*N*	Average	Standard deviation	Minimum	Q1	Median	Q3	Maximum
S3 A1	20	0.9016	0.1933	0.6648	0.7723	0.8651	0.9654	1.5343
S3 A2	20	1.0274	0.2193	0.7108	0.8060	1.0343	1.2096	1.4195
S3 B1	20	0.9726	0.1312	0.8473	0.8895	0.9405	1.0026	1.4151
S3 B2	20	0.9628	0.1357	0.8224	0.8597	0.9386	1.0052	1.3536
S3 D	20	1.3981	0.2027	0.9821	1.2878	1.3515	1.5804	1.8019
S3 T	20	1.1830	0.2019	0.9041	1.0132	1.1431	1.3218	1.6730

## Data Availability

All used data is within the paper.
